# The predictive efficacy of hypoechoic lesion in ultrasound for prostate cancer in Chinese people: five-year experience in a moderated 10-core transperineal prostate biopsy procedure

**DOI:** 10.18632/oncotarget.18342

**Published:** 2017-06-02

**Authors:** Tian Yang, Limin Zhang, Yixin Chen, Yehua Cai, Haowen Jiang, Qiang Ding

**Affiliations:** ^1^ Department of Urology, Huashan Hospital, Fudan University, Shanghai, China; ^2^ Department of Urology, Huashan North Hospital, Fudan University, Shanghai, China; ^3^ Fudan Institute of Urology, Huashan Hospital, Fudan University, Shanghai, China; ^4^ Department of Ultrasonography, Huashan Hospital, Fudan University, Shanghai, China

**Keywords:** PSA, transperineal prostate biopsy, prostate cancer, transrectal ultrasound, hypoechoic lesion

## Abstract

We aim to investigate the predictive efficacy of hypoechoic lesion for prostate cancer at different levels of serum PSA in the procedure of transrectal ultrasound guided 10-core trans-perineal prostate biopsy (TP-PBx). In this study, we collected clinical parameters involving age, digital rectal examination (DRE), PSA, prostate volume, pathological diagnosis, Gleason score, novel Gleason group, and numbers of positive cores from 856 patients who had elevated level of PSA above 4 ng/ml or susceptible nodule of prostate gland in DRE received the moderated 10-core TP-PBx procedure. There were 481 cases (56.2%) with no visible lesion of hypoechoic nodule in transrectal ultrasound (TRUS) and 375 cases (43.8%) with the hypoechoic lesion. The total cancer detection rate is 45.56%. The predictive efficacy of hypoechoic lesion for prostate cancer varies among different PSA intervals. For PSA groups of 0–4, 4–10, 10–20, 20–100, > 100 ng/ml, the Youden’s indexes are 0.3483, 0.3506, 0.3941, 0.2795 and 0.8667, respectively. Besides, the visible lesions are inclined to be detected in patients with higher Gleason score. We concluded that the hypoechoic lesions in TRUS could improve the predictive accuracy for diagnosing prostate cancer and present different predictive efficacy in the respective PSA intervals. Besides, it was probably associated with more aggressive clinical significance.

## INTRODUCTION

Prostate cancer (PCa) is one of the most frequently diagnosed malignant tumors and the second cause of cancer death among men worldwide [1]. The American Cancer Society estimates that in 2011, 240,890 men were diagnosed with PCa and 33,720 men died of it in United States [2]. The incidence of PCa was once relatively rare in Asia. In 1991, an epidemiological study reported a 26-fold higher rate of PCa in American than in Chinese men with an intermediate rate in Chinese-American men [3]. However, in the past few years, the prevalence of PCa has been increasing in China with the annual percentage change of 12.6%, highest among all types of male cancer from 2000 to 2011 [4–5]. In 2015, it is estimated that nearly 60,300 new PCa cases and 26,600 cancer deaths related to PCa occur in China [5]. Factors including earlier and frequent prostate-specific antigen (PSA) screening, improved skills of biopsy and western diet habit may explain this situation [5].

TRUS technology has become a mainstay of many image guided prostate interventions, including prostate biopsy, brachytherapy, cryotherapy, and high-intensity focused US [6]. Today PSA-based screening of asymptomatic men has resulted in the adaptation of TRUS biopsy as the standard of care when prostate biopsy is used to identify prostate cancer [6]. Since the introduction of the TRUS probe by Watanabe et al. [7, 8] and the development of the diagnostic procedure first applied in 1981 by Holm and Gammelgard [9], the value of TRUS for the detection and evaluation of PCa has been reported [10, 11]. However, the diagnostic efficacy of ultrasound for PCa has been a matter of debate in the past few decades [12, 13].

Although TRUS owns the disadvantage of poor specificity of abnormalities and the difficulty on the differentiation of tumor and adjacent benign tissues [14], it improves visualization of prostate lesions and is routinely used by most urologists for the diagnosis and staging of localized prostate cancer. Nowadays, it is widely accepted that 60–70% of prostate cancers are hypoechoic, and about 30–40% are isoechoic or nonvisible [15, 16]. Prostate cancer originating in hyperechoic lesions are extremely rare with an incidence of 1% to 1.5% [17–20].Only a few cases were described in the literature which were related to desmoplastic reaction of the prostate cancer [21].

The early detection of prostate cancer, especially the cases with clinical significance, is surely the keystone for the disease control. High levels of serum PSA, abnormal digital rectal examination (DRE) findings and hypoechoic lesions found during TRUS are the typical signs considered to be suspected for PCa, and TRUS guided prostate biopsy is recommended subsequently. In China, due to the regional disequilibrium in the social economic support and the accessibility of high standard healthcare, PSA test and conventional ultrasound-guided prostate biopsy will remain to be the major diagnostic tools for prostate cancer for quite a period of time.

In this study, we included different PSA intervals and scaled hypoechoic lesions as different types of the region of interest (ROI) in order to evaluate the validity of hypoechoic lesion in ultrasound as a predictive factor for PCa in Chinese patients.

## RESULTS

Among 856 cases who met the criteria, 481 (56.2%) cases didn’t have visible lesion of hypoechoic nodule in TRUS and 375 (43.8%) cases had hypoechoic lesion. None of the cases had hyperechoic nodule. The total cancer detection rate was 45.56%. The detection rate of hypoechoic lesion in TURS was 68.53%. The baseline characteristics of study population were shown in Table 1. A higher age, elevated PSA, smaller prostate volume and malignant pathological diagnosis were all significantly associated with hypoechoic lesions. Multivariate analysis of factors predicting PCa was shown in Table 2. Hypoechoic lesion (OR = 2.989, 95% CI = 2.018–4.427, *p* < 0.001) was also found independently associated with PCa.

**Table 1:** Baseline clinical characteristics of study population

	No Visible lesion of hypoechoic nodule in TRUS ^†^ (No. of cases = 481)	Hypoechoic lesion in TRUS (No. of cases = 375)	Significance
**Age (yrs)**			
Mean ± SD^‡^	68.88 ± 8.56	71.09 ± 8.39	*P* = 0.00
Median (range interquartile)	69 (13)	71 (12)	
**PSA§ (ng/ml)**			
Mean ± SD	25.65 ± 98.69	92.07 ± 247.83	*P* = 0.00
Median (range interquartile)	11.59 (12.04)	18.04 (50.22)	
DRE^*^			*P* = 0.00
Negative	450	199	
Unilateral nodule	28	109	
Bilateral nodule	3	67	
**Prostate volume (ml)**			
Mean ± SD	55.65 ± 25.49	46.67 ± 23.19	*P* = 0.00
**Pathological diagnosis**			*P* = 0.00
Malignant	133	257	
Benign	348	118	
**Gleason score**			
6	51	33	
3 + 4 = 7	24	49	
4 + 3 = 7	29	73	
8	19	47	
9 – 10	10	55	

†TRUS: transrectal ultrasound.

‡SD: standard deviation.

§PSA: prostate specific antigen.

*DRE: digital rectal examination.

**Table 2:** Multivariate analysis of factors predicting prostate cancer

	Odds Ratio	*P*	Lower CI^†^	Upper CI
Age	1.076	0.00	1.051	1.102
PSA	1.044	0.00	1.032	1.056
Prostate volume	0.954	0.00	0.944	0.964
Hypoechoic lesion	2.989	0.00	2.018	4.427

†CI: confidence interval.

Binary logistic regression analysis was conducted to compare the predictive accuracy for predicting models with and without hypoechoic lesion. When hypoechoic lesion was included in the regression model, the -2 likelihood ratio, Cox & Snell R^2^ and Nagelkerke R^2^ were 693.55, 0.423 and 0.565, respectively. When hypoechoic lesion was excluded in the regression model, the -2 likelihood ratio, Cox & Snell R^2^ and Nagelkerke R^2^ were 723.52, 0.402, and 0.537, respectively. This result showed that hypoechoic lesion could improve the predictive accuracy for diagnosing PCa.

The proportion of different PSA intervals in all patients and in patients with PCa was shown in Figure 1. The sensitivity, specificity, positive predict value (PPV) and negative predict value (NPV) of hypoechoic lesion for PCa in all patients were 65.90%, 74.68%, 68.53% and 72.50%. The predictive efficacy of hypoechoic lesion for PCa varied among different PSA intervals. The sensitivity, specificity, PPV and NPV were 90.91%, 44.83%, 38.46%, 92.86% when PSA was less than 4 ng/ml. When PSA ranged from 4–10 ng/ml, the sensitivity, specificity, PPV, NPV were respectively 58.18%, 76.88%, 41.03%, and 78.35%. In the group with PSA 10–20 ng/ml, those four values were 59.41%, 80.00%, 64.52%, and 76.30%. In the group with PSA 20–100 ng/ml, the 4 values were 60.81%, 67.14%, 79.64%, and 44.76%. In the last interval of PSA more than 100 ng/ml, the 4 values were 86.67%, 100%, 65.00%, 23.08% (Table 3). The Youden’s indexes of the five PSA groups were 0.3483, 0.3506, 0.3941, 0.2795 and 0.8667, respectively. The comparison of detecting cancer by different ROI types with respective PSA intervals was presented in Table 4. In patients with PSA > 20 ng/ml, the detection rate was significantly associated with ROI groups.

**Figure 1:** (**A**) The proportion of different PSA intervals in total patients (*n* = 856). (**B**) The proportion of different PSA intervals in patients with PCa (*n* = 390).

**Table 3:** The predictive efficacy of hypoechoic lesion for prostate cancer among different PSA intervals

PSA intervals (ng/ml)		Cancer	Non-cancer	Sensitivity (%)	Specificity (%)	PPV^†^ (%)	NPV^‡^ (%)	*P* value
0–4	no visible lesion	1	13	90.91	44.83	38.46	92.86	0.03
	hypoechoic lesion	10	16					
4–10	no visible lesion	23	153	58.18	76.88	41.03	78.35	0.00
	hypoechoic lesion	32	46					
10–20	no visible lesion	41	132	59.41	80.00	64.52	76.30	0.00
	hypoechoic lesion	60	33					
20–100	no visible lesion	58	47	60.81	67.14	79.64	44.76	0.00
	hypoechoic lesion	90	23					
>100	no visible lesion	10	3	86.67	100	65.00	23.08	0.00
	hypoechoic lesion	65	0					

†PPV: positive predict value.

‡NPV: negative predict value.

**Table 4:** The comparison of detecting cancer by different ROI^†^ types with respective PSA intervals

PSA intervals (ng/ml)		ROI = 1 (*N* = 175)		ROI = 2 (*N* = 41)		ROI = 3 (*N* = 40)		ROI = 4 (*N* = 87)		ROI = 5 (*N* = 32)		*P* value
		cases	Detection rate	cases	Detection rate	cases	Detection rate	cases	Detection rate	cases	Detection rate	
0–10	Cancer	29	35.80%	0	0	2	100%	4	66.67%	7	63.64%	> 0.05
	Non-cancer	52		4		0		2		4		
10–20	Cancer	25	51.02%	12	66.67%	5	83.33%	10	90.90%	8	88.89%	> 0.05
	Non-cancer	24		6		1		1		1		
> 20	Cancer	27	60.00%	18	94.74%	32	100%	67	95,71%	11	91.67%	< 0.01
	Non-cancer	18		1		0		3		1		

†ROI: region of interest.

The relationship between hypoechoic lesion and Gleason scores in different PSA intervals was shown in Table 5. As we can see from the table, the hypoechoic lesions were inclined to be detected in patients with higher Gleason score. In patients with PSA > 20 ng/ml, hypoechoic lesions were significantly associated with Gleason Group.

**Table 5:** The relationship between hypoechoic lesion and Gleason scores in different PSA intervals

PSA intervals (ng/ml)		Gleason Group 1	Gleason Group 2	Gleason Group 3	Gleason Group 4	Gleason Group 5	*P* value
0–10	no visible lesion	14	3	5	2	0	> 0.05
	hypoechoic lesion	12	10	15	2	3	
10–20	no visible lesion	16	8	11	6	0	> 0.05
	hypoechoic lesion	14	12	16	10	8	
> 20	no visible lesion	21	13	13	11	10	< 0.01
	hypoechoic lesion	7	27	42	35	44	

## DISCUSSION

Prostate cancer is a very common malignant disease and its incidence increases with age. Nowadays, TRUS-guided biopsy is still the only accurate preoperative method for early diagnosis of prostate cancer [22]. Besides having a great importance in guiding the needle direction for prostate biopsy, TRUS allows the visualization of suspected focal lesions of prostate cancer [23, 24]. A study [25] revealed prostate cancer was detected in 25.5% with a hypoechoic lesion through transrectal ultrasound directed prostatic biopsies. Another study [26] found that biopsy samples taken when a prostate lesion is identified by TRUS are almost twice as likely to show cancer than when no lesion is visible, These two studies concluded that the search for and targeting of hypoechoic lesions on TRUS remains important for PCa diagnosis. Hypoechoic lesions can also be detected in other diseases including granulomatous prostatitis, prostatic infarct and lymphoma [27]. Therefore, it is necessary to perform a biopsy on hypoechoic lesions. In our study, 68.53% of the patients with hypoechoic lesions were diagnosed as PCa by 10-core TP-PBx. The detection rate was a little higher than the recent reports with the detection rate of about 62.9%–67.2% by the same biopsy method [28, 29]. The reasons may attribute to our larger population and different skills of urologists in different medical centers.

In order to investigate the relationship between PCa and hypoechoic lesions further, we reclassified the patients according to different PSA intervals. We found that hypoechoic lesions were significantly associated with the diagnosis of PCa in all the PSA intervals and had the highest predictive efficacy in patients with PSA > 100 ng/ml, as expected, followed by PSA 10–20, PSA 4–10, PSA < 4 and PSA 20–100 ng/ml groups. When we divided ultrasound results into different ROI types, similar results were also found in patients with PSA > 20 ng/ml, which confirmed the diagnostic value of hypoechoic lesion. Few studies examined the utility of hypoechoic lesion, a TRUS-related indicator of potentially prostate cancer, as a risk factor in different PSA intervals. Our study may provide a new dimension into the diagnostic value of hypoechoic lesion in prostate cancer. More confirmatory studies are needed in the future.

In our study, patients who had hypoechoic lesions on TURS had a higher Gleason Grade group than those who didn’t, especially for patients with PSA > 20 ng/ml. This result was consensus with other studies [30]. Ellis and Brawer [31] also confirmed that Gleason score was independent of ultrasound findings. Newton et al. [32] summarized that prostate volume is inversely associated with high-grade PCa as well as extraprostatic extension and positive surgical margins. We also found that patients with hypoechoic lesions tended to have smaller prostate volume.

The multi-parametric MRI is another important examination for the diagnosis and treatment of PCa, especially targeted prostate biopsy [33]. Compared to TRUS, multi-parametric MRI owns better tissue resolution. It can compare the relative signal intensity within the prostate and identify lesions with poorly defined or irregular borders, which may have a higher suspicion of cancer [6, 34]. Therefore, multi-parametric MRI has a higher accuracy in the detection of clinically significant PCa than TRUS [35]. However, unlike ultrasound, the process of MRI examination is static and urologists can’t get dynamic images of prostate through MRI. Besides, ultrasound owns almost no contraindications and has a less economic burden on patients, which is more suitable and popular in China.

Recently, the use of transperineal template biopsies of the prostate (TTBP) has attracted many urologists and several studies have been published in the literature to explore this procedure [36, 37]. TTBP is a more invasive procedure than TRUS guided biopsy. An average of 58 core biopsies per patient is considered acceptable for mapping TTBP [38]. A study compared the diagnostic accuracy of TRUS-guided prostate biopsy and TTBP in 124 patients who were attributed a favorable risk prostate cancer status based on previous transrectal ultrasound guided biopsy and who were considering a policy of active surveillance, showing that repeat transrectal ultrasound biopsy failed to detect up to 80% of clinically important cancers detected by TTBP [39]. Another study also indicated that TTBP could find an upgrade of Gleason score in more than 20% of patients who were diagnosed with prostate cancer by previous transrectal biopsies [40]. Although TTBP has a higher diagnostic value than conventional 10-core TRUS-guided prostatic biopsies, the average number of core biopsies taken in a mapping TTBP is significantly high and patients are more likely to suffer a degree of pain and discomfort after TTBP [41]. Besides, the complication of acute urinary retention is reported in about 17% of patients who underwent TTBP [42–44]. Therefore, it remains controversial whether TTBP can completely replace TRUS-guided biopsy. In our study, we proved that 10-core TP-PBx would also have a considerable diagnostic value when we divided patients into different ROI types and PSA intervals.

Therefore, we concluded in our study that the hypoechoic lesions in TRUS could improve the predictive accuracy for diagnosing prostate cancer and present different predictive efficacy in the respective PSA intervals. Besides, it was probably associated with more aggressive clinical significance.

## MATERIALS AND METHODS

### Study population

From 2011.1.1 to 2015.12.15, patients who had elevated level of PSA above 4 ng/ml or susceptible nodule of prostate gland in DRE received the moderated 10-core TP-PBx procedure with the collaboration between the urologist and the physician of ultrasound medicine. Patients were informed consent. We consecutively collected 882 cases. Nine cases were excluded because of the failure of Gleason scoring and 17 cases were excluded because of the missing of PSA value. Thus, 856 cases met the criteria and were enrolled.

### Instruments

The major instruments used for the TP-PBx procedure were ultrasound scanner EUB-7500 (Hitachi) and Max-Core disposable core biopsy instrument (Bard Peripheral Vascular, Inc.)

### Method

Clinical parameters involving age, DRE, PSA, prostate volume, pathological diagnosis, Gleason score, novel Gleason group, and numbers of positive cores were documented for each patient. Patients were divided into several subgroups, according to different PSA level and transrectal ultrasound findings.

A moderated 10-core TP-PBx procedure was applied in the research. We divided the prostate gland into 10 areas in the sonographic image including the apex, base, body, posterolateral of peripheral zone and the transitional zone in lobes on both sides (Figure 2). Hypoechoic nodules were detected as the region of interest (ROI). When the ROI was located in a certain area, the free-hand targeted biopsy procedure was performed. Otherwise, the systematic TP-PBx was performed.

**Figure 2:** Different sections of prostate and the location of prostate biopsy in 10-core TP-PBx procedure (**A**) Transverse section. (**B**) Sagittal section. (**C**) Coronal section. (A. 1. apex of peripheral zone in left lobe; 2. base of peripheral zone in left lobe; 3. transitional zone in left lobe; 4. body of peripheral zone in left lobe; 5. posterolateral of peripheral zone in left lobe; 6. apex of peripheral zone in right lobe; 7. base of peripheral zone in right lobe; 8. transitional zone in right lobe; 9. body of peripheral zone in right lobe; 10. posterolateral of peripheral zone in right lobe). TZ: transitional zone.

The biopsy specimen was formalin-fixed and paraffin-embedded. The sections were stained with hematoxylin and eosin. Two pathologists independently evaluated the sections and delivered Gleason scores to the cases of PCa, which would be judged by a superior pathologist when two pathologists made the different diagnosis. According to the novel prostate cancer grading system [45], we reclassified the patients by the new five grades based on the revised original Gleason score: group 1 (Gleason score ≤ 6), group 2 (Gleason score 3 + 4 = 7), group 3 (Gleason score 4 + 3 = 7), group 4 (Gleason score 8), and group 5 (Gleason score 9–10).

The ROI type was divided into 5 types according to the tumor stage of PCa partially. ROI type I: small nodule occupying less than the half volume of peripheral zone (PZ) in the unilateral lobe; ROI type II: the volume of the hypoechoic lesion larger than the half and less than the whole PZ in unilateral lobe; ROI type III: the lesion infiltrating the whole PZ area of one lobe; ROI type IV: the diffused invasion in bilateral lobes; ROI type V: the incidence of multiple hypoechoic lesions in the whole prostate gland.

Cox & Snell R^2^, Nagelkerke R^2^ and -2 likelihood ratio were used to evaluate the goodness of fit of binary logistic regression model. Higher Cox & Snell R^2^ and Nagelkerke R^2^ and a lower -2 likelihood ratio indicated a better goodness of fit. PPV, NPV and Youden’s index were used to evaluate the predictive efficacy of hypoechoic lesion in predicting PCa. PPV and NPV were defined as the proportions of positive and negative results in diagnostic tests that are true positive and true negative results, respectively. PPV reflected the possibility of PCa in patients who had hypoechoic lesion in ultrasound and NPV reflected the possibility of non-PCa in patients in patients who didn’t have hypoechoic lesion. Youden’s index was defined as sensitivity plus specificity minus one. PPV, NPV and Youden’s index were all indexes reflecting the performance of a diagnostic test. The higher the value of these indexes, the better the predictive efficacy.

Statistics analysis was conducted with the software of SPSS v20.0 (IBM Corp. U.S.A.). Continuous variables were expressed as either the mean ± standard deviation or the median. Categorical variables were reported as the number of occurrences and frequency. The student *t*-test was used to compare the means of continuous variables between groups. Chi-square test was used to compare categorical variables. Variables that showed significant differences were included in a multivariate logistic regression analysis. Two tail *p* values of < 0.05 were considered statistically significant.

There remained several limitations in our study. First, though the entire sample size of our study was not small, few patients had certain ROI type or Gleason Group in some of the PSA interval groups, which made it difficult and meaningless to analyze the diagnostic efficacy of hypoechoic lesions on TRUS. Secondly, besides hypoechoic lesion, the blood flow signal could also provide evidence in the detection of PCa. In our study, we didn’t carry out the blood signal examination of ultrasound, which needs further investigation. Thirdly, this is a prospective study from single institute, which might lead to selection bias. Our study can only partly represent the Chinese population, especially population from southeast part of China. Fourthly, we didn’t focus on the prognostic value of hypoechoic lesions in the current study. A long-time follow-up will be carried out to measure its value for evaluation of PCa progression.

## Abbreviations

PSA: prostate specific antigen
TP-PBx: trans-perineal prostate biopsy
DRE: digital rectal examination
TRUS: transrectal ultrasound
MRI: magnetic resonance image
PCa: prostate cancer
ROI: region of interest
SD: standard deviation
CI: confidence interval
PPV: positive predict value
NPV: negative predict value
TTBP: transperineal template biopsies of the prostate
TZ: transitional zone
